The article "Performance Related Factors Are the Main Determinants of the von Willebrand Factor Response to Exhaustive Physical Exercise" was published in 2014. Journal: PLoS One.

# Performance Related Factors Are the Main Determinants of the von Willebrand Factor Response to Exhaustive Physical Exercise

**DOI:** 10.1371/journal.pone.0091687

**Published:** 2014-03-13

**Authors:** Janine E. van Loon, Michelle A. H. Sonneveld, Stephan F. E. Praet, Moniek P. M. de Maat, Frank W. G. Leebeek

**Affiliations:** 1 Department of Haematology, Erasmus University Medical Center, Rotterdam, the Netherlands; 2 Department of Neurology, Erasmus University Medical Center, Rotterdam, the Netherlands; 3 Department of Rehabilitation Medicine, Erasmus University Medical Center, Rotterdam, the Netherlands; National Cerebral and Cardiovascular Center, Japan

## Abstract

**Background:**

Physical stress triggers the endothelium to release von Willebrand Factor (VWF) from the Weibel Palade bodies. Since VWF is a risk factor for arterial thrombosis, it is of great interest to discover determinants of VWF response to physical stress. We aimed to determine the main mediators of the VWF increase by exhaustive physical exercise.

**Methods:**

105 healthy individuals (18–35 years) were included in this study. Each participant performed an incremental exhaustive exercise test on a cycle ergometer. Respiratory gas exchange measurements were obtained while cardiac function was continuously monitored. Blood was collected at baseline and directly after exhaustion. VWF antigen (VWF:Ag) levels, VWF collagen binding (VWF:CB) levels, ADAMTS13 activity and common variations in Syntaxin Binding Protein-5 (*STXBP5,* rs1039084 and rs9399599), Syntaxin-2 (*STX2,* rs7978987) and VWF (promoter, rs7965413) were determined.

**Results:**

The median VWF:Ag level at baseline was 0.94 IU/mL [IQR 0.8–1.1] and increased with 47% [IQR 25–73] after exhaustive exercise to a median maximum VWF:Ag of 1.38 IU/mL [IQR 1.1–1.8] (p<0.0001). VWF:CB levels and ADAMTS13 activity both also increased after exhaustive exercise (median increase 43% and 12%, both p<0.0001). The strongest determinants of the VWF:Ag level increase are performance related (p<0.0001). We observed a gender difference in VWF:Ag response to exercise (females 1.2 IU/mL; males 1.7 IU/mL, p = 0.001), which was associated by a difference in performance. Genetic variations in *STXBP5*, *STX2* and the VWF promoter were not associated with VWF:Ag levels at baseline nor with the VWF:Ag increase.

**Conclusions:**

VWF:Ag levels strongly increase upon exhaustive exercise and this increase is strongly determined by physical fitness level and the intensity of the exercise, while there is no clear effect of genetic variation in *STXBP5*, *STX2* and the VWF promoter.

## Introduction

Blood coagulation changes in response to physical exercise [1]–[6]. One of the major players in blood coagulation is von Willebrand factor (VWF), a multifunctional glycoprotein that initiates primary haemostasis. Ultralarge very active VWF multimers are cleaved by *A Disintegrin and Metalloprotease with ThromboSpondin motif repeats 13* (ADAMTS13) into smaller, less prothrombotic forms. It is well known that levels of VWF increase steeply upon intense physical exercise [7]. To date it is not fully understood which mediators, both non-genetic and genetic, affect VWF response to stress. However, it is of great interest to discover new determinants of the excretion mechanism of VWF molecules, since high VWF levels have been associated with venous thrombosis [8] and arterial thrombosis [9]–[11].

VWF is mainly synthesized by endothelial cells and marks endothelial cell activation [12], [13]. The majority of the freshly synthesized VWF molecules are constitutively released into the circulation. A small part of especially large VWF multimers − harbouring the greatest haemostatic potential − is stored in Weibel Palade Bodies of endothelial cells [14]–[17]. Numerous agonists initiate the release from these storage granules, including hypoxia, epinephrine, histamine, thrombin, fibrin, and vasopressin [18], [19].

Plasma VWF levels have a wide biological variation, since numerous lifestyle factors, environmental factors, and genetic factors continuously influence VWF levels in the circulation [19]. Previous studies among human twins have demonstrated that more than half of the variability in VWF levels is caused by genetic variations in the genome [20], [21]. The most important genetic determinant is ABO blood group [22]. In addition, recently six new genetic loci have been discovered using a hypothesis-free approach with genome-wide association studies [23]. Two of the newly identified genetic loci, Syntaxin Binding Protein-5 (*STXBP5*) and Syntaxin-2 (*STX2*), are of specific interest, since their encoding proteins interact with SNARE complex proteins, such as SNAP23 and syntaxin-4, which have been shown to be involved in Weibel Palade Body (WPB) exocytosis, a well-known mechanism for the secretion of VWF molecules by endothelial cells [24]. Another genetic modulator is the VWF promoter in which four single nucleotide polymorphisms (SNPs) have been identified, that are associated with VWF levels [25], [26].

We aimed to identify important mediators, including lifestyle factors, environmental factors, and common genetic variations in the *STXBP5*, *STX2* and VWF promoter genes, of VWF response to incremental exhaustive exercise in a large group of young healthy individuals.

## Materials and Methods

### Ethics Statement

The study was approved by the medical ethical committee at Erasmus University Medical Center and written informed consent was obtained from all participants at inclusion.

### Study participants

For the “RESPOnse” (Role of SNARE protein genes in the regulation of von Willebrand Factor concentration and other coagulation factors) study, we included 105 healthy individuals, who were between 18 to 35 years of age and of North-European ancestry. Exclusion criteria were known cardiovascular risk factors, including hypertension, hypercholesterolemia, diabetes, obesity (BMI > 30 kg/m^2^), and a positive family history of cardiovascular disease. In addition, participants never had a thrombotic event or coagulation disorder, were non-smokers, had no known malignancies, no liver or renal dysfunction, did not use medication that may influence VWF levels and were not pregnant. Oral contraceptives use was allowed in this study. Subjects were requested to abstain from caffeinated and alcoholic beverages twelve hours prior to the test and to avoid heavy or high-intensity physical exercise and sports activities on the day of the test.

### Baseline measurements

At baseline, all patients received a questionnaire on current health status and physical condition. We measured weight using a calibrated digital scale (SECA GmbH & co, model 861) and height using a wall mounted telescopic height rod (SECA GmbH & co, model 220). Blood pressure was measured in an upright sitting position with a calibrated sphygmanometer (Welch Allyn, model Maxi-Stabil 3) and left upper-arm adjusted cuff size (WelchAllyn, FlexiPort reusable blood pressure cuff). Also, before the start of the cycle ergometer test, we performed a rest electrocardiogram (ECG) to exclude abnormalities in electric conduction through the heart, arrhythmias etc. All participants declared to be in good health and none of them had medical contra-indications for participation in the study.

### Cycle ergometer maximal test

Each participant performed an incremental exercise test until exhaustion, performed on a cycle ergometer (Ergoline, ER800, Lode, the Netherlands) using a linearly increasing (12 or 18.5 W min-1) ramp protocol. These slopes were chosen to achieve exhaustion within 8–12 minutes as recommended by Zhang et al [27]. Participants started with a warming-up phase of 4 minutes without resistance. They were instructed to pedal at a frequency between 60 and 80 rotations per minute (rpm). The loaded phase was terminated when pedalling frequency dropped below 60 rpm and was followed by cooling-down for at least 2 minutes.

Cardiac function was monitored using a 12-lead electrocardiogram with heart rate (HR) being recorded continuously. Respiratory gas exchange measurements were performed continuously by using a computerized metabolic cart (Oxycon Pro, Carefusion, the Netherlands) that was calibrated before each test. Maximal whole-body oxygen uptake capacity was defined in the present study as VO_2_ remaining unchanged or increasing less than 1 ml/min/kg for 30 sec or more despite an increment in work load [28]. VO_2_ is the capacity to transport and use oxygen during exercise and is a measure for physical fitness. The ventilatory threshold (VT1) was determined by an increase in ventilation (Ve)/VO_2_ but without a concomitant increase in Ve/VCO_2_. The ventilatory threshold represents the moment at which metabolism changes from aerobic to anaerobic. Two experienced exercise physiologists reviewed the plots averaged over 30 sec of the Ve/VO_2_ and Ve/VCO_2_ and determined VT1 values. In case of disagreement, the opinion of a third investigator was sought. The metabolic equivalent (METs) score is calculated by the VO2 max and VO2 VT1 values (1 MET  =  3.5 ml/min/kg VO2). A METs score (calculated by the VO2 max) above 10 represents activities associated with significant exertion. A METs score calculated by the VO2 VT1 represents the intensity to sustain activities for 1 hour and is a measurement of the physical fitness of an individual. The power output (W) was assessed to establish the workload capacity of the participant. Power output is dependent on physical fitness, but also on talent. Finally, maximum respiratory exchange ratio (RER) at peak power output was determined. The RER is a ratio between the amount of carbon dioxide (CO_2_) exhaled and the amount of oxygen (O2) inhaled per breath. Together with the maximum achieved heart rate as percentage of age-predicted heart rate (i.e. 208-0.7*age) [29], the maximum RER is a measure for the intensity of the test.

### Blood sampling

Venous blood was drawn from the forearm before and directly after exhaustion (within 1 minute) via a cannula in the antecubital vein using a Vacutainer system (Becton-Dickinson, Plymouth, UK). The first 2 ml of blood was discarded at every time point. Blood for coagulation measurements was collected in 3.2% trisodium citrate (9:1 vol/vol). Citrated blood was centrifuged within 1 hour at 3500 rpm for 10 min at 4°C. Plasma was additionally centrifuged at 14 000 rpm at room temperature and stored in aliquots at −80°C. For DNA isolation we stored the buffy coats of the remaining citrated blood at −20°C until use. Genomic DNA was isolated according to standard salting-out procedures and stored at 4°C for genetic analysis.

### Laboratory measurements

VWF antigen (VWF:Ag) was determined with an in-house ELISA with polyclonal rabbit anti-human VWF antibodies and horseradish peroxidase conjugated anti-human VWF antibodies (DakoCytomation, Glostrop, Denmark) for catching and tagging, respectively.

VWF collagen binding (VWF:CB) was determined with an in-house ELISA using collagen bovine antibodies and horseradish peroxidase conjugated anti-human VWF antibodies (DakoCytomation, Glostrop, Denmark) for catching and tagging, respectively.

ADAMTS13 activity was measured by a Fluorescence Resonance Energy Transfer Substrate (FRETS) assay using a fluorescent VWF peptide consisting of 73 amino acids (FRETS-VWF73). Plates were read with BioTek’s microplate reader (BioTek). The intra-assay coefficients of variation for VWF:Ag, VWF:CB and ADAMTS13 were 1.9%, 4.5% and 3.6%, respectively. The inter-assay coefficients of variation for VWF:Ag, VWF:CB and ADAMTS13 were 8.3%, 7.9% and 7.5%, respectively.

### Genotyping

The STXBP5 gene spans 182 kbps and is located in the q24 region of chromosome 6. Initially, we obtained data from the International HapMap project (phase II November 2008 http://www.hapmap.org) on the linkage disequilibrium (LD) pattern and selected haplotype-tagging single-nucleotide polymorphisms (ht-SNPs) using Haploview software (version 3.11; www.broad.mit.edu/mpg/haploview/index/php). For the *STXBP5* and *STX2* genes blocks of haplotypes with a frequency of ≥ 3% were defined in order to select these ht-SNPs. We took potential functionality into consideration by preferentially selecting non-synonymous ht-SNPs or SNPs that are located in known regulatory elements. We considered only SNPs that were present in a Caucasian population. Of these ht-SNPs, three were significantly associated with VWF:Ag levels in our previous study among young patients with arterial thrombosis and healthy controls [30]. Therefore, we selected and genotyped only these three SNPs in *STXBP5* (rs1039084 and rs9399599) and in *STX2* (rs7978987) for our current study. The polymorphisms in *STXBP5*, rs1039084 and rs9399599, are in high linkage disequilibrium with rs9390459, which had the highest genome wide significance level for VWF plasma levels in the meta-analysis of the CHARGE consortium (D’ = 1.00, R^2^ = 0.87 for rs9399599 and D’ =  0.96, R^2^ = 0.86 for rs1039084) (phase II November 2008 http://www.hapmap.org). Also, rs7978987 in *STX2* had a highly significant P value of 3.82×10^−11^ in this meta-analysis[23].

The gene encoding VWF is approximately 180 kb in length, contains 52 exons and is located on chromosome 12. Four SNPs in this gene have been identified, which are in strong linkage disequilibrium and segregate as two haplotypes [25], [31]. We have selected and genotyped one of these SNP’s (rs7965413).

Genotyping was done using Custom TaqMan Genotyping Assays (Applied Biosystems, Foster City, CA, USA). Endpoint fluorescence was measured on the ABI 7900HT instrument (Applied Biosystems, Foster City, CA, USA) and clustered according to genotype using SDS 2.1 software (Applied Biosystems, Foster City, CA, USA). Genotyping was successful for each SNP in on average 97% of all subjects.

### Statistical Analysis

Data on baseline characteristics are presented as means and standard deviations for continuous variables and as counts and percentages for categorical data. Since VWF:Ag levels were skewed, these data were natural logarithmically transformed (lnVWF:Ag) and presented as median and interquartile range (IQR). Mann-Whitney tests were used for unpaired two-group comparisons of non-parametric data.

The association between baseline characteristics and performance related determinants with lnVWF:Ag increase were assessed with linear regression models. Logistic regression was used to assess the relationship between VWF:Ag response and baseline characteristics, using VWF:Ag response as categorical variable. VWF:Ag increase was divided into two categories: low response with a VWF:Ag increase below the median (<0.40 IU/mL) and high response with a VWF:Ag increase above the median (≥ 0.40 IU/mL). Gender differences in performance-related determinants were assessed with univariate analysis of variance (ANOVA). The power output and the VO_2_ were adjusted for weight and presented as the value per kg.

Allele frequencies of the VWF polymorphisms were calculated by genotype counting. For each SNP, the deviation from the Hardy-Weinberg equilibrium was tested by means of a Chi-squared test with one degree of freedom. We used linear regression analyses with additive genetic models to determine the association between genetic variations in VWF and lnVWF:Ag levels. We had a power of 0.80 to detect a difference of 0.2 between carriers of the minor allele and carriers of the common allele, assuming a minor allele frequency of 0.40. Beta-coefficients represent the increase in lnVWF:Ag levels per coded allele. Statistical analyses were performed with SPSS for Windows, version 20.0 (SPSS Inc, Chicago, USA). A two-sided value of p<0.05 was considered statistically significant.

## Results

In the current study, 105 healthy individuals were included. Baseline characteristics are shown in table 1. The mean age was 24 years and 61% were female. Blood pressure (mean 114/70 mmHg) and BMI (mean 23 kg/m^2^) were within the normal range. Of all subjects, 86 (82%) used alcoholic beverages. Of all female participants, 33 women (52%) used oral contraceptives, seven women (11%) had an intra-uterine device (Mirena®), and two women (3%) had a Nuva ring®.

**Table 1:** Baseline characteristics.

	N = 105
**Age (years)**	24.3±4.4
**Female sex, N (%)**	64 (61%)
**Systolic blood pressure (mmHg)**	114±12
**Diastolic blood pressure (mmHg)**	70±9
**Heart rate (bpm)**	76±10
**BMI (kg/m^2^)**	23±2
**Oral contraceptives (% of total women)**	33 (52%)
**Blood group O, N (%)**	54 (51%)
**METs score (max)**	12.4±2.4
**METs score (VT1)**	8.6±1.9
**VWF:Ag baseline (IU/mL), median (IQR)**	0.94 (0.77–1.12)
**VWF:Ag maximum (IU/mL), median (IQR)**	1.38 (1.10–1.84)
**VWF:Ag absolute increase (IU/mL), median (IQR)**	0.40 (0.23–0.70)
**VWF:Ag relative increase (%), median (IQR)**	47 (25–73)
**VWF:CB baseline (IU/mL), median (IQR)**	0.93 (0.75–1.17)
**VWF:CB maximum (IU/mL), median (IQR)**	1.36 (1.11–1.68)
**VWF:CB absolute increase (IU/mL), median (IQR)**	0.37 (0.17–0.67)
**VWF:CB relative increase (%), median (IQR)**	43 (19–69)
**ADAMTS13 baseline (U/ml), median (IQR)**	1.28 (1.11–1.42)
**ADAMTS13 maximum (U/ml), median (IQR)**	1.46 (1.24–1.58)
**ADAMTS13 absolute increase (U/ml), median (IQR)**	0.15 (0.07–0.24)
**ADAMTS13 relative increase (%), median (IQR)**	12 (6–19)
**VWF:CB/VWF:Ag ratio baseline, median (IQR)**	1.00 (0.91–1.10)
**VWF:CB/VWF:Ag ratio maximum, median (IQR)**	0.96 (0.89–1.05)

Summary statistics for continuous variables are presented as mean ± standard deviation. Categorical data are summarized as percentages. VWF:Ag, VWF:CB and ADAMTS13 levels and the VWF:CB/VWF:Ag ratio are presented as median and interquartile range (IQR).

The median VWF:Ag level at baseline was 0.94 IU/mL and increased with 47% after exhaustive exercise to a median maximum VWF:Ag of 1.38 IU/mL (p<0.0001) (Table 1, Figure 1). The median VWF:CB level at baseline was comparable with the VWF:Ag level, 0.93 IU/mL, and increased with 43% to a median maximum of 1.36 IU/mL (p<0.0001). The absolute increase in VWF:Ag and VWF:CB levels was highly correlated (R 0.81, p<0.0001). The VWF:CB/VWF:Ag ratio was 1.00 at baseline and was decreasing to 0.96 at maximum exercise. ADAMTS13 levels also increased after exhaustive exercise with 12% (Table 1, Figure 1). There was no correlation between the absolute increase in VWF:Ag level and ADAMTS13 (R 0.06, p = 0.57).

**Figure 1:** Levels (U/ml) of VWF:Ag, VWF:CB, ADAMTS13 and the ratio VWF:CB/VWF:Ag at baseline and maximum. P values represents the difference between baseline and maximum levels.

Baseline characteristics were not associated with baseline VWF:Ag levels (table 2). As expected, blood group non-O was associated with higher baseline VWF:Ag levels (geometric mean of VWF:Ag for blood group O: 0.82±0.03 IU/mL and for non-O: 1.08±0.05 IU/mL). Sex, systolic blood pressure, and diastolic blood pressure were significantly associated with the VWF:Ag level response (Table 2 and Figure 2). Alcohol consumption, defined as any amount of glasses per week, was borderline significantly associated with a lower VWF:Ag response (p = 0.06). The strongest determinant was sex. In a multivariate model including sex, blood pressure, and alcohol consumption, only sex remained significantly associated with VWF:Ag levels (beta-coefficient for males 0.79 [95% CI 0.52;1.06], p<0.0001).

**Figure 2:** Association between baseline characteristics and VWF:Ag response defined by the Odds ratio. VWF:Ag increase divided into two categories: low response with a VWF:Ag increase below the median (<0.40 IU/ml) and high response with a VWF:Ag increase above the median (≥0.40 IU/ml).

**Table 2:** Association between baseline characteristics and VWF:Ag levels.

	Baseline VWF:Ag levels		Absolute VWF:Ag increase	
	Beta-coefficient [95% CI]	P-value	Beta-coefficient [95% CI]	P-value
**Age**	0.01 [–0.004; 0.02]	0.18	–0.03 [–0.06;0.01]	0.14
**Male sex**	–0.02 [–0.14;0.10]	0.73	0.79 [0.54;1.04]	< 0.0001
**Systolic blood pressure**	0.001 [–0.01;0.01]	0.93	0.02 [0.003;0.03]	0.02
**Diastolic blood pressure**	–0.004 [–0.11;0.002]	0.21	0.02 [0.001;0.03]	0.04
**BMI**	–0.002 [–0.03;0.02]	0.90	0.02 [–0.05;0.08]	0.60
**Alcohol consumption**	–0.10 [–0.26;0.05]	0.18	–0.36 [–0.74;0.01]	0.06
**Blood group non-O**	0.28 [0.17;0.39]	< 0.0001	–0.10 [–0.39;0.19]	0.48
**Oral contraceptives**	–0.04 [–0.21;0.14]	0.67	–0.23 [–0.59;0.14]	0.22

Univariate linear regression analysis, beta-coefficient represents the increase of lnVWF:Ag levels with 95% confidence interval per unit increase of the selected variable.

At baseline, we observed no difference in VWF:Ag levels between males and females (median [IQR]: females 0.95 IU/mL [0.78;1.12] and males 0.91 IU/mL [0.74;1.11], p = 0.50). At exhaustion, males had significantly higher VWF:Ag levels than females (females 1.22 IU/mL [1.06;1.58] and males 1.66 IU/mL [1.24;2.05], p = 0.001). OAC use was not associated with the VWF:Ag level response to exercise.

Next, we investigated the association between performance related determinants and the VWF:Ag response (table 3A). All performance-related determinants were significantly associated with the increase in VWF:Ag levels, but not with the baseline VWF:Ag levels. The strongest performance related determinants (p<0.0001) were the peak power output per kg bodyweight, the ratio between the power output at the ventilatory threshold and the peak power output in Watt, VO_2_ peak per kg and the maximum RER at peak power output. Physical fitness, as represented by the VO_2_ VT1/max and power output VT1/max, was negatively associated with the VWF:Ag increase. In addition, a multivariate regression was performed. However, strong multicolinearity was observed between all performance-related variables. Therefore, we selected variables that showed the least correlation with each other for the multivariate model. To this end, we used two models with different combinations of variables. Nevertheless, multicolinearity could not be excluded completely, whereby the results of the multivariate regression analysis should still be interpreted with care. Next, we added sex to model I and model II, which resulted in the loss of the significant association between sex and VWF:Ag increase (Model I: β = 0.27 [95% CI –0.04;0.58], p = 0.09; model II: β = 0.23 [95% CI –0.84;0.54], p = 0.15). Additionally, when stratifying for sex the association between performance related determinants and the increase in VWF:Ag levels remained. In table 3B the performance-related values are presented for males and females separately. Physical fitness (VO_2_ VT1/max and power output VT1/max) was slightly higher in females than in males. The intensity of the test and the endurance of the participant, as represented by the VO2 peak, peak power output, and the maximum RER, were higher in males than in females. There was no difference in test duration between males and females. When excluding women with oral contraceptives the results of the study did not change.

**Table 3:** Performance-related determinants of VWF:Ag increase and mean differences between males and females.

	A			B		
	Univariate	Multivariate Model I	Multivariate Model II	Males	Females	
	β [95% CI]	β [95% CI]	β [95% CI]	N = 41	N = 64	P-value
**Peak Power Output per kg**	0.57 [0.42;0.72]*		0.51 [0.36;0.65]*	4.4±0.1	3.4±0.1	< 0.0001
**Watts per kg VT1**	0.42 [0.17;0.66]†			2.8±0.1	2.3±0.1	< 0.0001
**Watts VT1/ Watts max**	–2.57 [–3.95; –1.20]*	–1.02 [–2.36;0.33]		63±1	67±1	0.04
**VO_2_ peak per kg**	0.05 [0.03;0.06]*	0.04 [0.03;0.06]*		50.2±1.0	39.2±0.8	< 0.0001
**VO_2_ VT1 per kg**	0.03 [0.01;0.05]†			33.9±0.9	27.9±0.7	< 0.0001
**VO_2_ VT1/VO_2_ peak**	–2.14 [–3.55; –0.72]†		–0.41 [–1.66;0.83]	68±2	72±1	0.051
**Max Respiratory Exchange Ratio**	3.75 [2.01;5.49]*	2.52 [0.79;4.25]†	2.49 [0.90;4.07]†	1.18±0.01	1.13±0.01	0.001
**Test duration**	0.09 [0.03–0.15]†			18.1±0.3	18.2±0.3	0.90

Linear regression analysis with natural log VWF:Ag as dependent. Beta-coefficient represents the increase in lnVWF:Ag per unit increase of the selected variable.* p<0.0001, † p<0.01.

A Performance related determinants of VWF:Ag increase in the total population.

B Gender differences in performance-related determinants.

Finally, we investigated the association between genetic variations in *STXBP5*, *STX2* and VWF promoter on VWF:Ag response to exercise (table 4). There was no significant association between genetic variations and VWF:Ag levels at baseline, at exhaustion, nor an association with the absolute VWF:Ag increase. Also, ABO blood group, the most important genetic determinant of VWF:Ag levels, was not associated with the VWF:Ag level response to exercise. There was also no significant difference in the association between VWF increase and genetic variation between individuals with blood group O and individuals with blood group non-O (data not shown).

**Table 4:** VWF:Ag levels per genotype of polymorphisms in *STXBP5*, *STX2* and VWF promoter.

	N	Baseline (IU/mL)	Exhaustion (IU/mL)	Absolute difference (IU/mL)
**rs1039084 (STXBP5)**				
**GG**	33	0.94±0.06	1.45±0.08	0.52±0.06
**AG**	44	1.02±0.05	1.56±0.07	0.54±0.05
**AA**	25	0.96±0.06	1.42±0.10	0.46±0.06
**P for trend**		0.44	0.44	0.67
**rs9399599 (STXBP5)**				
**AA**	32	0.89±0.06	1.40±0.09	0.51±0.06
**AT**	45	1.05±0.05	1.59±0.07	0.54±0.05
**TT**	25	0.96±0.06	1.41±0.10	0.45± 0.06
**P for trend**		0.11	0.18	0.56
**rs7978987 (STX2)**				
**GG**	48	0.98±0.05	1.43±0.07	0.45±0.05
**AG**	45	0.98±0.05	1.55±0.07	0.57±0.05
**AA**	12	0.94±0.09	1.42±0.14	0.47±0.09
**P for trend**		0.94	0.43	0.18
**rs7965413 (VWF promoter)**				
**AA**	47	1.01±0.05	1.48±0.07	0.47±0.05
**AG**	40	0.94±0.05	1.43±0.08	0.49±0.05
**GG**	13	1.03±0.09	1.61±0.13	0.58±0.09
**P for trend**		0.55	0.50	0.55

## Discussion

In this study among 105 healthy young subjects, VWF:Ag levels increased significantly upon incremental exhaustive exercise (mean METs score (max) >10) with a median increase of 47%. The VWF:Ag response was highly variable and was strongly dependent on performance-related and physical fitness-related determinants. Neither baseline characteristics nor the studied genetic determinants of VWF:Ag levels affected the extent of VWF:Ag response to physical exercise.

VWF:CB levels increased after exhaustive exercise in the same proportion as VWF:Ag levels. ADAMTS13 levels at baseline were in the high normal range. This study included young and healthy individuals and a previous study also showed higher levels in young individuals [3]. ADAMTS13 levels increased after exhaustion, although it was to a lower extent than VWF levels. A previous study showed similar results as ADAMTS13 increased after exercise in patients with von Willebrand disease type 2B [3]. However, in another study in healthy individuals there was no difference in ADAMTS13 between baseline and immediately after exercise [3], [5]. In addition, ADAMTS13 decreased after infusion of desmopressin, which induces a release of large VWF multimers into the circulation, in healthy individuals [32]. However, all these studies included only low number of patients.

As the average maximal achieved heart rate as a percentage of age-predicted maximum heart rate was 97±6%, together with a plateauing of oxygen uptake and a mean RER of 1.15±0.08, our test protocol can be considered as an exhaustive cycle ergometer test in our subjects [33], [34].

In our study, VWF:Ag levels increased significantly upon physical exercise. This was comparable with a previous study which showed a significant increase in VWF:Ag levels post exercise and 15 minutes after exercise [35]. We found a higher increase in VWF:Ag response upon exercise in males compared with females. After stratifying for sex, the association between the performance related determinants and the VWF:Ag increase did not change. This indicates that the role of physical fitness and the intensity of the test on VWF:Ag response upon exercise is independent of sex. Women taking oral contraceptives were not excluded for this study. As oral contraceptives have effects on coagulation factors [36] this could have influenced our results. However, no differences were found when excluding those women and additionally no significant differences were found between women using oral contraceptives and women without (data not shown).

In our study, the VWF:Ag levels increase upon exercise was the highest in individuals with the lowest physical fitness, although this was not significant after multivariate analysis, and in individuals with the most intensive exercise. Intensive physical exercise is associated with more recruitment of capillaries in the muscle and additionally an increase in vascular conductance in muscle composed predominantly of fast-twitch oxidative (type IIa) and fast-twitch glycolytic (type IIb) fibers [37]. This results in more endothelial exposure to shear stress and adrenergic stimulation, which may explain the increased release of VWF upon exercise. The highest VWF:Ag response in individuals with the lowest physical fitness underlines the hypothesis that frequent physical exercise has a positive effect on cardiovascular risk. This is in contrast with a previous study which showed no difference in VWF:Ag increase upon exercise between resistance trained and untrained individuals [35]. However, in this study only a small number of individuals were included (N = 20). For a long time it has been anticipated that regular physical exercise has a favourable effect on many biological mechanisms, thereby improving health and fitness. Regular physical exercise is associated with a decreased all-cause mortality and with a reduced cardiovascular risk [38]. The positive effects of physical exercise on cardiovascular disease development may be induced by alterations in haemostasis that lead to a hypocoagulable state. This hypocoagulable state is achieved by a compensatory exhaustion of platelets in physically active individuals and underlines the beneficial effects of exercise on long-term prevention of cardiovascular disease [39]. In our study, the baseline VWF:Ag levels were not associated with physical fitness or intensity of the test. This observation is in line with previous findings that showed that levels of coagulation factor VII (FVII), VWF, and FVIII at rest were similar in professional athletes and controls [40]. There are multiple factors which could have influenced our results, including the type of sport and the training status of the participants, which are known to influence e.g. capillary density and in vivo endothelial function in skeletal muscle. However, the majority of our subjects participated in recreational type of sports activities and can be regarded as a representative sample of healthy active individuals.

*STXBP5* and *STX2* are two novel genetic loci that have been associated with VWF:Ag levels in the general population [23]. In addition, genetic variation within these genes affects VWF:Ag levels in young patients with a first event of arterial thrombosis [30]. Considering the involvement of the *STXBP5* and *STX2* encoding proteins in the regulated secretion of VWF molecules, our hypothesis was that genetic variants within these genes would affect the release of VWF molecules, but not the steady state levels, which are determined by the constitutive pathway. To this end, we included young individuals below the age of 35 years to exclude the presence of extensive atherosclerosis, which is related to endothelial dysfunction and consequent higher VWF:Ag levels. Their baseline VWF:Ag levels therefore represent a steady state situation. To provoke release of VWF molecules from Weibel Palade Bodies in our study, all participants performed exhaustive physical exercise, which induces beta-adrenergic receptor activation [41] and subsequent endothelial cell activation. Genetic variation in *STXBP5* and *STX2* was not associated with VWF:Ag levels at baseline, though we had sufficient power to detect the previously observed effect of these genetic variants. The VWF:Ag increase upon exercise was also not affected by genetic variation in *STXBP5* and *STX2*. This finding was in contrast to our hypothesis.

In addition, we genotyped a common variation in the VWF promoter gene. Previous studies have shown an association between this genetic variation and VWF:Ag levels at baseline [25], [31]. However, other studies have failed to show an effect of this polymorphism on VWF levels under normal conditions [42]–[44]. Despite the fact that the influence of genetic variation in the VWF promoter on VWF levels has never been studied in arterial thrombosis or at stress before, we hypothesized that a genetic variation in this gene would affect the expression of VWF at physical exercise resulting in a difference in VWF plasma levels. In our study, we could not find a significant association between baseline VWF:Ag levels and genetic variations in the VWF promoter gene, probably caused by a relatively small study population. Furthermore, the VWF:Ag increase upon exercise was also not associated with the VWF promoter. This suggests that, in contrast to our hypothesis, the VWF release is not depending on genetic variations in the VWF promoter at exhaustive physical exercise.

The negative results of the influence of genetic variation on VWF increase may be caused by the fact that genetic variations in *STXBP5* and *STX2* may not be involved in WPB exocytosis. In addition, VWF is also stored in alpha-granules of platelets and the contribution of platelet VWF to plasma levels upon exercise is not known [45]. Therefore, VWF release from platelet alpha-granules during exercise cannot be excluded and might explain the negative results of the role of genetic variations involved in Weibel Palade Body exocytosis. Furthermore, we observed that the VWF:Ag increase was highly variable and strongly dependent on physical fitness and the intensity of the exercise performed. Consequently, the effect of environmental factors may have been stronger than the genetic effect.

Another important genetic determinant of VWF:Ag levels is blood group [46]. Individuals with blood group O have 25% lower VWF:Ag levels than individuals with blood group non-O, because the presence of blood group A and B antigens on VWF molecules leads to a decreased clearance of VWF molecules [47]. Furthermore, blood group non-O has been associated with an increased risk of CHD [48]–[50]. Ribeiro et al. observed that males with blood group non-O (N = 8) had higher post-exercise VWF:Ag levels than males with blood group O (N = 8), although the rise of VWF:Ag was not statistically significantly different between the groups [51]. In our study, subjects with blood group non-O had higher levels at exhaustion (median [IQR], 1.60 IU/mL [1.2–2.0]), than subjects with blood group O (1.29 IU/mL [1.1–1.6], p = 0.03). However, blood group was not associated with the VWF:Ag increase upon exercise (0.49 IU/mL [0.2–0.8] in non-O versus 0.46 [0.2–0.7] in O, p = 0.34). Assuming that exercise induces the release of VWF molecules from its storage granules and the clearance does not change during exercise, it was expected that subjects with blood group O and subjects with blood group non-O had a similar increase after exercise. In this study, we only included young healthy individuals and therefore the results of the study cannot be extrapolated to the older population. However, those individuals were included to exclude the presence of extensive atherosclerosis which represents a steady state situation.

In conclusion, we have shown in a large and homogeneous group of young healthy individuals that VWF:Ag levels increase strongly upon exhaustive physical exercise and is primarily dependent on physical fitness and the intensity of the exercise performed. Genetic variations in *STXBP5*, *STX2* and VWF promoter that have previously been identified as important genetic determinants of VWF:Ag levels, were not associated with the VWF:Ag response to physical exercise. Also, ABO blood group, the most important genetic determinant of VWF:Ag levels was not associated with the VWF:Ag increase. These findings suggest that environmental factors may be more important than genetic factors in determining the VWF:Ag response to stress.
